# Decoding the Mechanism behind the Pathogenesis of the Focal Segmental Glomerulosclerosis

This article has been retracted.

**DOI:** 10.1155/2022/1941038

**Published:** 2022-04-19

**Authors:** Xiao Zhu, Liping Tang, Jingxin Mao, Yasir Hameed, Jingyu Zhang, Ning Li, Danny Wu, Yongmei Huang, Chen Li

**Affiliations:** ^1^School of Laboratory Medicine, Hangzhou Medical College, Hangzhou 310053, China; ^2^The Eighth Medical Center, Chinese PLA General Hospital, Beijing 100091, China; ^3^College of Pharmaceutical Sciences, Southwest University, Chongqing 400715, China; ^4^Department of Biochemistry and Biotechnology, The Islamia University of Bahawalpur, Bahawalpur 63100, Pakistan; ^5^Southern Marine Science and Engineering Guangdong Laboratory (Zhanjiang), Guangdong Medical University, Zhanjiang 524024, China; ^6^Department of Biology, Chemistry, Pharmacy, Free University of Berlin, Berlin 14195, Germany

## Abstract

Focal segmental glomerulosclerosis (FSGS) is a chronic glomerular disease associated with podocyte injury which is named after the pathologic features of the kidney. The aim of this study is to decode the key changes in gene expression and regulatory network involved in the formation of FSGS. Integrated network analysis included Gene Expression Omnibus (GEO) datasets to identify differentially expressed genes (DEGs) between FSGS patients and healthy donors. Bioinformatics analysis was used to identify the roles of the DEGs and included the development of protein-protein interaction (PPI) networks, Gene Ontology (GO), and the Kyoto Encyclopedia of Genes and Genomes (KEGG) pathway enrichment analyses, and the key modules were assured. The expression levels of DEGs were validated using the additional dataset. Eventually, transcription factors and ceRNA networks were established to illuminate the regulatory relationships in the formation of FSGS. 1130 DEGs including 475 upregulated genes and 655 downregulated genes with functional enrichment analysis were determined. Further analysis uncovered that the validated hub genes were defined as candidate genes, including Complement C3a Receptor 1 (C3AR1), C-C Motif Chemokine Receptor 1(CCR1), C-X3-C Motif Chemokine Ligand 1 (CX3CL1), Melatonin Receptor 1A (MTNR1A), and Purinergic Receptor P2Y13 (P2RY13). More importantly, we identified transcription factors and mRNA-miRNA-lncRNA regulatory networks associated with the candidate genes. The candidate genes and regulatory networks discovered in this study can help to comprehend the molecular mechanism of FSGS and supply potential targets for the diagnosis and therapy of FSGS.

## 1. Introduction

Focal segmental glomerulosclerosis (FSGS) is a common glomerular disease, accounting for 40% of adult cases and 20% of children, with the major cause of the steroid-resistant nephrotic syndrome and end-stage renal disease [1]. The incidence of the disease has gradually increased in recent years and the prognosis is relatively poor, with 50% of patients gradually progressing to end-stage renal disease within 5 to 10 years, accounting for about 20% of dialysis patients [2]. In 1970, the international children's kidney disease research collaboration formally proposed FSGS as a separate clinicopathological syndrome [3]. The main pathological manifestations of FSGS are focal and segmental sclerosis of the affected glomeruli, corresponding tubular atrophy, and interstitial fibrosis [4]. FSGS is clinically characterized by varying degrees of proteinuria, which may be accompanied by nephrotic syndromes such as microscopic hematuria, hypertension, or impaired tubular function, and is prone to complications such as infection and deep vein thrombosis [5]. The pathogenesis of FSGS is not fully understood and is currently thought to be caused by a range of podocyte injury factors, including circulating factor-mediated podocyte injury; podocyte gene mutations; viral infections such as human immunodeficiency virus, Epstein-Barr virus, and cytomegalovirus; nephrotoxic drug injuries such as heroin, alpha interferon, rapamycin, and calcium-regulated phosphatase inhibitors; and dysplastic factors such as very low birth weight, congenital nephrogenic unitopia with compensatory hypertrophy, and unilateral renal hypoplasia [6]. In recent years, there has been an increasing trend in renal biopsy detection rates of FSGS reported around the world, and the incidence of FSGS varies by region worldwide [7]. In the Americas, FSGS has become a major pathological type of glomerular disease; in the Middle East, South Asia, and Europe, the prevalence is high; and in other parts of Asia, the prevalence is increasing year by year, although it is not a major pathological type [8].

The noncoding RNAs (ncRNAs) serve as functional regulators that are transcribed from DNA but not translated into proteins [9]. The miRNAs, circRNAs, and lncRNAs are involved in the ncRNA epigenetic regulation. Generally, ncRNAs function to regulate gene expression at the transcriptional and posttranscriptional level. In the last decade, ncRNA has drawn more and more consideration in the chronic kidney disease from both bench and clinic sides [10]. Previous studies have disclosed the emerging roles of ncRNA and related message RNA (mRNA) in the development of various kidney diseases, including chronic kidney disease [11]. Chen et al. revealed that retinoic acid receptor responder protein 1, which is mainly restricted to podocytes, upregulates in the glomerular of the chronic nephrosis patients. Inversely, lower Rarres1 improved Adriamycin-induced nephropathy in the inducible RARRES1 knockdown mice [12]. By using a rodent FSGS model induced by Adriamycin, Qi et al. suggested that miR-150 inhibitor exerts protective effect on the glomerular via ameliorating renal fibrosis and inflammation [13]. The ncRNAs also serve as a diagnostic biomarker for FSGS [14] and can value the progression of chronic kidney disease [15]. Nevertheless, few studies have clarified systematically the regulatory network and mechanism in the pathogenesis of focal segmental glomerulosclerosis.

For the clear knowledge of the biomarkers, we screened microarray data of mRNAs in glomeruli samples from FSGS patients and healthy donors in the current study. After identification and validation, hub different expression genes (DFGs), transcription factors (TFs), and competing endogenous RNA (ceRNA) network were reconstructed, respectively, which were exploited to illustrate the regulatory mechanism. Our output discriminated FSGS-related genes with high credibility in the patients and empowered a more comprehensive approach to identify diagnosis and therapeutic targets for FSGS.

## 2. Materials and Methods

### 2.1. Data Processing and Screening of Differentially Expressed Genes (DEGs)

The overall study design is illustrated in Figure 1. The expression profiling datasets GSE108109, GSE104066, and GSE104948, organized from Homo sapiens, were obtained from the publicly available Gene Expression Omnibus (GEO) [16]. These datasets were based on the GPL19983 [HuGene-2_1-st] Affymetrix Human Gene 2.1 ST Array [HuGene21st_Hs_ENTREZG_19.0.0] platform or GPL22945 [HG-U133_Plus_2] Affymetrix Human Genome U133 Plus 2.0 Array [CDF: Brainarray HGU133Plus2_Hs_ENTREZG_v19] platform (Table 1). The interactive web tool GEO2R is employed to screen of differentially expressed genes (DEGs) from selected datasets (GSE108109 and GSE104066) individually [17]. The DEGs between FSGS samples and living donor samples under the following threshold were retained, an adjusted *P* value < 0.05 and a ∣log fold change | >1, as the mRNA were decoded for the following analysis.

### 2.2. DEG Functional and Pathway Enrichment Analysis

Gene Ontology (GO) function [18] and Kyoto Encyclopedia of Genes and Genomes (KEGG) pathway enrichment [19] analysis of overlapping genes were analyzed by utilizing the Metascape, an online enrichment analysis tool for gene annotation [20]. Three categorized enrichments, biological process, cellular component, molecular function, are involved in the Gene Ontology (GO) functional enrichment. The adjusted *P* < 0.05 and an enriched gene count > 5 were set as criteria for significance for the identification of GO terms and KEGG pathways, with the top 20 terms visualized.

### 2.3. Integration of protein-protein interaction (PPI) network and identification of the most significant modules and hub genes

The Search Tool for the Retrieval of Interacting Genes (STRING) is a web tool to predict interactions between the proteins of candidate genes [21]. The shared DEGs were mapped to STRING to evaluate the interaction, and the PPI pairs that confidence score of *v* ≥ 0.9 were considered significant. Cytoscape software was used to visualize and construct PPI network [22]. The hub genes were identified by CytoHubba [23] with 5 chosen methods, degree method (Deg), density of maximum neighborhood component (DMNC), edge percolated component (EPC), maximum neighborhood component (MNC), and maximal clique centrality (MCC). To investigate more specific regulatory relationship of proteins, the molecular complex detection (MCODE) [24] was carried out to screen the crucial clustering modules in the PPI network with the default setting.

### 2.4. Validation of Hub Genes by Separated Datasets

To verify the robustness of hub genes, a separated dataset GSE104948 was utilized to validate the differential expression of these hub genes. GraphPad Prism software was used to calculate and generate bar plots.

### 2.5. Integration of Validated Hub Gene-Transcription Factor Network

Transcription factors (TF) are essential for the regulation of gene expression and are, as a consequence, found in all living organisms. NetworkAnalyst is an integrated platform for TFs-gene interaction in numerous species to identify the vital TFs with validated hub genes [25]. In addition, the ENCODE database that produced the TFs-gene network is included in the NetworkAnalyst. The validated hub gene-TF network was also visualized by Cytoscape.

### 2.6. The miRNA Prediction and Validated Hub Gene-miRNA Network Construction

The modulations between the miRNAs and 5 validated hub genes of FSGS were built by Cytoscape via 5 miRNA databases, namely, TargetScan [26], DIANA-microT [27], miRDB [28], miRWalk [29], and miRmap [30]. The overlapping miRNAs were involved in more than 3 databases selected as the predicted results.

### 2.7. The Associated lncRNA Prediction and ceRNA Network Construction

According to the regulatory relationship, lncRNAs can act as miRNA sponges, affecting their regulatory effect on mRNAs. The interactions between lncRNAs and miRNAs that are related to 5 validated hub genes were predicted by the starBase database [31]. Afterward, based on the acquired lncRNA-miRNA pairs, the competing endogenous RNA (ceRNA) network was mapped by bonding lncRNA-miRNA-mRNA pairs and visualized via the Cytoscape.

### 2.8. Statistical Analysis

SPSS 18.0 software was employed to perform statistical analysis. The significant differences between the two groups were evaluated by Student's *t*-test. Data are expressed as mean ± S.D. The *P* value < 0.05 was considered as significant. All authors take full responsibility for the integrity of the data.

## 3. Results

### 3.1. DEGs between the FSGS Patients and Living Donors

DEGs in the glomeruli tissues of patients with FSGS were identified compared with healthy donors. In total, it is reported in Figure 2(a), 624 upregulated and 764 downregulated genes were identified between FSGS patients and healthy donors in the GSE108109. Meanwhile, 494 upregulated and 702 downregulated genes were identified between FSGS patients and healthy donors in the GSE104066. Moreover, the top DEGs could discriminate between the patients with FSGS and the healthy donors in Figure 2(b). The intersection of upregulated genes or downregulated genes from two datasets (GSE108109 and GSE104066) is shown in the Venn diagram (Figure 2(c)); among these overlapping genes, 475 genes were upregulated genes and 655 genes were downregulated genes, and these consistently changed mRNAs were selected as overlapped genes for the next further analysis.

### 3.2. GO and KEGG Annotations of DEGs

The pathogenesis of FSGS is complicated, and comprehending the functions of the DEGs can indicate the novel bench studies and clinic treatments. Each part of GO enrichments is displayed in Figures 3(a)–3(c) (upregulated DEGs) and Figures 3(e)–3(g) (downregulated DEGs). For biological process (BP) enrichment analysis, the results showed that the upregulated DEGs strongly took part in the vasculature development, blood vessel development, positive regulation of cellular component movement, positive regulation of cell motility, and positive regulation of cell migration (Figure 3(a)). The downregulated genes were strongly involved in monocarboxylic acid metabolic process, alpha-amino acid metabolic process, cellular amino acid metabolic process, organic acid catabolic process, and alpha-amino acid catabolic process (Figure 3(e)). For cell component (CC) enrichment analysis, the present study showed that the upregulated DEGs were mainly involved in extracellular matrix, external encapsulating structure, side of membrane, collagen-containing extracellular matrix, and endocytic vesicle (Figure 3(b)). The downregulated DEGs mainly revolved in apical plasma membrane, apical part of the cell, brush border membrane, basolateral plasma membrane, and basal plasma membrane (Figure 3(f)). In addition, in the enrichment analysis of molecular function (MF), upregulated DEGs are significantly enriched in cell adhesion molecule binding, integrin binding, growth factor binding, protein homodimerization activity, and actin binding (Figure 3(c)). For downregulated DEGs, they significantly take part in sodium ion transmembrane transporter activity, solute-sodium symporter activity, butyrate-CoA ligase activity, secondary active transmembrane transporter activity, and bitter taste receptor activity (Figure 3(g)).

Moreover, the KEGG pathway enrichment analysis by upregulated DEGs and downregulated DEGs was listed, respectively. Among the pathways, AGE-RAGE signaling pathway in diabetic complications, cytokine-cytokine receptor interaction, Epstein-Barr virus infection, chemokine signaling pathway, and TNF signaling pathway are involved in the mechanism of upregulated DEGs (Figure 3(d)). On the side, downregulated DEGs were mainly enriched in drug metabolism-cytochrome P450, retinol metabolism, drug metabolism, metabolism of xenobiotics by cytochrome P450, and taste transduction (Figure 3(h)).

### 3.3. PPI Network Analysis, Most Significant Modules and Hub Gene Identification for Suggesting Therapy

To illustrate the PPI network of these overlapped DEGs, the analysis was constructed through the STRING platform and was visualized by Cytoscape (Figure 4). We totally found 820 paired interactions and 175 upregulated and 80 downregulated genes involved in this network (Supplementary file 1-2).

The subnetwork of genes acts crucial roles in the whole integrated networks. Module analysis on the PPI network through the molecular complex detection (MCODE) plugin revealed top 10 significant clusters, which are shown in Figure 5(a). Cluster 1 with the highest cluster score of 22 includes Apelin Receptor (APLNR), Complement C3a Receptor 1 (C3AR1), Complement C5a Receptor 1 (C5AR1), C-C Motif Chemokine Ligand 5 (CCL5), C-C Motif Chemokine Receptor 1 (CCR1), C-X3-C Motif Chemokine Ligand 1 (CX3CL1), C-X-C Motif Chemokine Ligand 16 (CXCL16), G Protein Subunit Gamma 2 (GNG2), G Protein Subunit Gamma 7 (GNG7), Kininogen 1 (KNG1), Melatonin Receptor 1A (MTNR1A), Purinergic Receptor P2Y13 (P2RY13), Prostaglandin E Receptor 3 (PTGER3), Sphingosine-1-Phosphate Receptor 4 (S1PR4), and bitter taste receptor family (TAS2R10, TAS2R14, TAS2R19, TAS2R20, TAS2R3, TAS2R31, TAS2R4, and TAS2R5). Additionally, the overlapped DEGs were imported into CytoHubba plugin of Cytoscape, which was used to screen out top 20 crucial genes through 5 different algorithms, including degree method (Deg), density of maximum neighborhood component (DMNC), edge percolated component (EPC), maximum neighborhood component (MNC), and maximal clique centrality (MCC). Subsequently, 14 common genes were selected by overlapping the 20 genes, as shown in Table 2; these 14 common genes are also involved in the gene cluster 1. To learn the tissues that these 14 genes express, we screened the database and the literature. The TAS2R family genes are excluded since the proteins that are encoded by these genes are specifically expressed in the taste receptor cells of the tongue and palate epithelia. Ultimately, C3AR1, C5AR1, CCR1, CX3CL1, CXCL16, MTNR1A, P2RY13, PTGER3, and S1PR4 are identified as the hub genes (Figure 5(b)).

### 3.4. Validation of Hub Gene Expression

All the 9 hub genes underwent expression validation in GSE104948 (GPL22945). GraphPad Prism was used to perform Student's *t*-test statistical analyses and draw boxplots (Figure 6). Consistent with our previous predictions, C3AR1, CCR1, CX3CL1, and P2RY13 were significantly upregulated in FSGS compared to living donors (*P* < 0.05), while MTNR1A was significantly downregulated in FSGS compared to the living donors (*P* < 0.05). However, PTGER3, S1PR4, C5AR1, and CXCL16 showed no significance between FSGS samples and healthy donors in dataset GSE104948 (GPL22945), which may be affected by the small sample size. As a result, we found that C3AR1, CCR1, CX3CL1, MTNR1A, and P2RY13 exhibited accordantly significant expression changes in these three datasets.

### 3.5. TF-Gene Interactions

In order to explore transcriptional signatures of the 5 validated hub genes, the TF-validated hub gene networks are found in Figure 7. The network covers 25 TF-validated hub gene pairs totally. CX3CL1 was modulated by 20 TFs, C3AR1 was modulated by 3 TFs, and MTNR1A was modulated by 2 TFs. No TFs regulate more than one validated hub genes in the network. There were no predicted TF of CCR1 and P2RY13.

### 3.6. Exploration of the miRNA-mRNA Network

The regulatory network that involved the predicted miRNA-validated hub gene pairs is shown in Figure 8, which revealed that one validated hub gene was modulated by multiple miRNAs. Subsequently, we obtained 57 target miRNAs of 5 validated hub genes and identified 58 mRNA-miRNA pairs. miRNA-6124 could affect mRNA CX3CL1 and CCR1 at the same time. No other miRNAs regulate more than one validated hub genes in the network.

### 3.7. Construction of the lncRNA-Associated ceRNA Network

To identify correlations in the ceRNA network, coexpressed lncRNA-miRNA pairs and circRNA-miRNA pairs were screened. Afterward, 18 lncRNAs all associated with target miRNAs were obtained. Finally, the lncRNA-miRNA-mRNA ceRNA networks were constructed, respectively, including 4 mRNAs, 11 miRNAs, and 18 lncRNAs (Figure 9). We observed that merely the upregulated mRNAs (P2RY13, CX3CL1, CCR1, and C3AR1) are involved in both ceRNA networks; there were no predicted lncRNAs of miRNAs that target MTNR1A which is downregulated in the FSGS.

## 4. Discussion

Although multiple factors are involved in the pathogenesis of FSGS, noteworthy primary FSGS is present in approximately 80% of cases [32]. Abundant evidence has confirmed that genetic factors play a vital part in the progression of FSGS; there are not only racial differences but also more than 18% of FSGS have familial aggregation [33]. Furthermore, mutations in the master effector gene take the leading role in the FSGS supposedly, which differs from other glomerular nephropathies [34]. Combined symptomatic therapy with hormone and cytotoxic drugs is most frequent in the FSGS, but the serious side effects caused by the high doses of hormone drugs are still inevitable [35]. Meanwhile, transplantation therapy involving endothelial progenitor cells and mesenchymal stem cells has received good achievements in animal experiments [36]. Blood purification is an emerging application for FSGS clinically, but large-scale controlled trials are still lacking [37]. Considering that the etiologies of the FSGS are not understood, the overall curative outcome is relatively poor compared with other pathological types.

As the rapid development of sequencing and microarray that are widely applied in clinical diagnosis and bench medicine, this contributes to the essential biomarker filtrations and discovers in the combat with the various diseases [38]. Booming genes have been reported to be associated with the incidence of FSGS, with the majority of mutations causing before adulthood [39]. The discovery of FSGS-associated genes can deepen our knowledge and also has implications for therapy to prevent unnecessary hormone and immunosuppressive application. Especially, genetic sequencing for the suspected colony with gene mutations should be performed at an early stage of FSGS. In addition, gene sequencing also can be applied for the next generation in the family genetic counseling [40]. Comprehensive bioinformatics means supported in an analysis of how critical genes vary; totally, 88 FSGS patients and 28 healthy donors from 3 studies were selected in the present study that was initiated to discover the diagnostic biomarkers and therapeutic targets for FSGS. Initially, we manually extracted and overlapped all the DFGs from GSE108109 and GSE104066 and identified 1130 DEGs, including 475 upregulated DEGs and 655 downregulated DEGs.

Then, we processed these up- and downregulated genes, respectively, for GO function and KEGG pathway enrichment analysis to clarify the role of these DEGs. The GO annotation demonstrated that upregulated DEGs in the FSGS were significantly enriched in vasculature development, blood vessel development, extracellular matrix, and cell adhesion molecule binding, which are consistent with previous evidence. Angiogenesis is the process of forming new blood vessels and requires the development and growth of endothelial cells which are the main cell type of the glomerulus. Leaky vessels, faulty blood vessels, and abnormal vessel growth play a role in the progression of FSGS [41]. The focal activation of parietal epithelial cells is initiated by loss of podocytes and forms cellular adhesions with the capillary tuft followingly [42]. FSGS is defined as the segmental or globular glomerulosclerosis due to the reduced number of podocytes and accumulation of extracellular matrix [43]. KEGG enrichment analysis revealed that AGE-RAGE is a significant signaling pathway; the receptor for advanced glycation end products (RAGE) was upregulated at the base of podocytes; especially, the endogenous secretory RAGE was highly detected in the serum of FSGS patients [44]. Kim and Dryer proved that *α*V*β*3-integrin and RAGE in podocytes act as coreceptors for soluble urokinase plasminogen activator receptor (suPAR) signaling and that elevated expression leads to poor outcomes in chronic nephrosis in the recent report [45]. Additionally, the previous results are in line with downregulated KEGG analysis which showed that retinol metabolism is a remarkable pathway. Circulating retinol-binding protein 4, which is bound to retinol in the bloodstream, is high in children with steroid-resistant nephrotic syndrome-FSGS than first episode nephrotic syndrome [46].

Fourteen overlapped hub genes include C3AR1, C5AR1, CCR1, CX3CL1, CXCL16, MTNR1A, P2RY13, PTGER3, S1PR4, TAS2R10, TAS2R19, TAS2R3, TAS2R4, and TAS2R5 which were identified by constructing the PPI network and weighing by CytoHubba and MCODE from Cytoscape. The training dataset (GSE104948) was used to verify the correlation between these overlapped hub genes and FSGS patients. We validated these data and came to the further conclusion that C3AR1, CCR1, CX3CL1, and P2RY13 are significantly high and MTNR1A is obviously low in the FSGS patients. In accordance with our findings, a recent report elucidated that the activation of complement in kidney cells with increased generation of C3 contributes to the induced podocyte injury in primary membranous nephropathy [47]. The emerging studies of chemokines and chemokine receptors showed a distinct perspective on the chronic nephropathy pandemic [48]. Theoretically, chemokines majorly act as a chemoattractant to guide the migration of leukocytes and immune cells in the respective anatomical locations [49]. Specifically, chemokines can effectively accelerate renal leukocyte trafficking and activation and subsequent local damage [50, 51]. Conclusively, various nephroses occur from the excessive infiltration of immune cells. BX471, the CCR1 antagonist, adequately weakened interstitial leukocyte accumulation in the murine FSGS model and the subsequent renal fibrosis [52]. It is worth mentioning that MRS2365 is a selective antagonist of the P2Y(13) receptor with the potential capacity to cure multiple allergic conditions [53]. Besides, melatonin affects the tubular via melatonin receptors (MTNRs) located in the kidney of mammals [54]. Huang et al. indicated that decreased MTNR1A occurs in the cytoplasm of tubular epithelial cells from experimental membranous nephropathy mice and blocking the MTNR1A receptor by luzindole causes further aggravating nephritis [55, 56]. These prior proofs are in accordance with our findings.

A wide number of studies have indicated that the dysfunction of transcription factors is related to the onset or progression of FSGS [57–60]. All the 25 transcription factors found in our study are the participants in the progress of diverse renal diseases. It is worth noting that ATF3, which was found in the urine exosomes of the rat kidney injury model, aggravated podocyte injury [61, 62]. Ebf1 contributed to the development and maturation of glomerular as well as podocyte via the mediation of COX-2 expression and calcineurin/NFAT pathway [63, 64]. The inducible expression of SMAD4 is a critical segment in the process of podocyte apoptosis in chronic kidney diseases, as well as the development of kidney diseases [65, 66]. We definitely concentrate on the potentiality of these transcription factors being novel drug targets for FSGS through epigenetic modulation.

FSGS is a heterogeneous group of glomerular disorders or podocytopathies, and accumulating studies indicated that dysregulation of microRNAs was involved in the process of the podocytes [67]. Upregulated expression of miR-378a-3p induced glomerular dysfunction in the proteinuric nephropathy, especially promoting podocyte effacement in the FSGS mammalian model [68]. Moreover, a comparative study pointed out that microRNAs in the circulating and urinary could act as potent biomarkers for diagnosis and also for therapy monitor [69]. Gebeshuber et al. reported that overexpressed miR-193a restrains the expression of the Wilms' tumor protein (WT1) and its target genes, which impairs the homeostasis of podocytes, and ultimately causes FSGS, as well as increased expression of miR-193a was also found in the FSGS patients [70]. Existing reports described that there are intricate interactions among diverse RNA molecules, such as protein-coding messenger RNAs and noncoding RNAs (circRNAs, lncRNAs, and miRNAs). Crosstalk RNA molecules cooperate to generate a dynamic regulatory network functioning as competitive endogenous RNAs (ceRNAs) [71]. However, limited literature reports the ceRNA network in the podocyte or FSGS, thus showing a bright prospect. The P38/C/EBP*β* pathway induced expression of long noncoding RNA LOC105374325, competitively binds miR-34c/miR-196a/b, and ulteriorly leads to increased levels of Bax and Bak in podocytes from individuals with FSGS [72]. In another study, circZNF609 caused podocyte injury in vivo and in vitro via decreasing miR-615-5p, WT1, and podocin expression [73]. Nevertheless, we are cautious of these competitive network analyses. To the best of our knowledge, there have been no studies on ceRNA networks in FSGS. In our study, ceRNA networks were built based on the interactions between lncRNA-miRNA and miRNA-mRNA. 18 lncRNA nodes, 11 miRNA nodes, and 4 mRNA nodes were included in the networks. Upon comprehensive analysis of the ceRNA network, some novel and crucial characteristics of FSGS were disclosed.

The potential limitations of this study need to be considered. First, three datasets contain different populations of FSGS patients and controls, which may implicate the results. Additionally, because the data we analyzed were obtained from public databases, further experiments are necessary to validate the findings.

## 5. Conclusion

In summary, these findings provide new perspectives into the pathogenesis of FSGS and might ascertain potential diagnostic and therapeutic approaches for the following studies. Further analysis is needed to investigate the molecular mechanisms by which the five key genes affect the prognosis of patients with FSGS.

## Figures and Tables

**Figure 1:** The workflow of the study design.

**Figure 2:** DEGs between FSGS patients and healthy donors from GSE104066 and GSE108109, respectively. (a) Volcano plots. (b) Heatmaps. (c) Venn diagrams indicate overlap of upregulated genes and downregulated DEGs, respectively.

**Figure 3:** The functional and pathway enrichment analysis of the overlap DEGs between the FSGS patients and healthy donors. (a) Molecular function, (b) biological process, (c) cellular component, and (d) KEGG of overlap upregulated genes. (e) Molecular function, (f) biological process, (g) cellular component, and (h) KEGG of overlap downregulated genes.

**Figure 4:** The PPI network of overlap DEGs between the FSGS patients and healthy donors.

**Figure 5:** Identification of the most significant modules and hub genes. (a) Top 10 modules of DEGs between the FSGS patients and healthy donors. The subclusters 1-10 were extracted from PPI networks. (b) 14 hub genes were identified by overlapping the first 20 genes in the 5 classification methods of CytoHubba.

**Figure 6:** The mRNA expression of the 9 hub genes was validated by the GSE104948 dataset.

**Figure 7:** The network of validated hub gene-TF. The red round rectangle nodes are the validated hub genes, and yellow V-shaped nodes are the TFs.

**Figure 8:** Network of predicted miRNAs, showing relationships between 57 miRNAs and 5 validated hub genes (mRNAs). The red rectangle nodes are the validated hub genes (mRNAs), and the green ellipse nodes are miRNAs.

**Figure 9:** Interaction of RNAs in the FSGS-associated ceRNA network. The red rectangle nodes are the validated hub genes (mRNAs), the green ellipse nodes are the miRNAs, and the blue diamond nodes are the lncRNAs.

**Table 1:** The summary of included microarray sets.

Series	Platform	Sample size	FSGS		Glomeruli	Species
			FSGS	Living donor		
GSE108109 [74]	GPL19983	111	30	6	36	Homo sapiens
GSE104066 [75]	GPL19983	76	48	6	54	Homo sapiens
GSE104948 [74]	GPL22945	71	10	16	26	Homo sapiens

**Table 2:** The top hub genes ranking in the CytoHubba.

Rank methods in CytoHubba					Shared top hub genes
Degree	DMNC	EPC	MCC	MNC	
KNG1	APLNR	GNG2	APLNR	GNG2	TAS2R5
GNG2	CX3CL1	KNG1	CX3CL1	GNG7	TAS2R4
GNG7	TAS2R10	C3AR1	TAS2R10	KNG1	TAS2R3
C3AR1	TAS2R3	GNG7	TAS2R3	S1PR4	TAS2R19
EGF	TAS2R4	TAS2R10	TAS2R4	APLNR	TAS2R10
S1PR4	TAS2R5	TAS2R14	TAS2R5	CX3CL1	S1PR4
CCL5	CXCL16	C5AR1	CXCL16	TAS2R10	PTGER3
APLNR	CCR1	TAS2R19	CCR1	TAS2R3	P2RY13
CX3CL1	C3AR1	CCL5	C3AR1	TAS2R4	MTNR1A
TAS2R10	MTNR1A	S1PR4	MTNR1A	TAS2R5	CXCL16
TAS2R3	P2RY13	TAS2R31	P2RY13	CXCL16	CX3CL1
TAS2R4	C5AR1	CXCL16	C5AR1	CCR1	CCR1
TAS2R5	PTGER3	P2RY13	PTGER3	C3AR1	C5AR1
CXCL16	TAS2R19	TAS2R3	TAS2R19	MTNR1A	C3AR1
CCR1	TAS2R31	CX3CL1	TAS2R31	P2RY13	
MTNR1A	TAS2R20	CCR1	TAS2R20	C5AR1	
P2RY13	TAS2R14	MTNR1A	TAS2R14	PTGER3	
C5AR1	CCL5	TAS2R4	CCL5	TAS2R19	
PTGER3	S1PR4	PTGER3	S1PR4	TAS2R31	
TAS2R19	ACTN1	TAS2R5	ACTN1	TAS2R20	

## Data Availability

The expression profiling datasets GSE108109, GSE104066, and GSE104948, organized from Homo sapiens, were obtained from the publicly available Gene Expression Omnibus (GEO). These datasets were based on the GPL19983 [HuGene-2_1-st] Affymetrix Human Gene 2.1 ST Array [HuGene21st_Hs_ENTREZG_19.0.0] platform or GPL22945 [HG-U133_Plus_2] Affymetrix Human Genome U133 Plus 2.0 Array [CDF: Brainarray HGU133Plus2_Hs_ENTREZG_v19] platform.

## Supplementary Materials

Supplementary 1 Supplementary file 1: the 820 paired interactions in the PPI network.

Supplementary 2 Supplementary file 2: the regulations of genes in the PPI network.

## References

[1] D'Agati V. D., Kaskel F. J., Falk R. J. (2011). Focal segmental glomerulosclerosis. *New England Journal of Medicine*.

[2] Jacobs-Cachá C., Vergara A., García-Carro C. (2021). Challenges in primary focal segmental glomerulosclerosis diagnosis: from the diagnostic algorithm to novel biomarkers. *Clinical Kidney Journal.*.

[3] Sethi S., Glassock R. J., Fervenza F. C. (2015). Focal segmental glomerulosclerosis: towards a better understanding for the practicing nephrologist. *Nephrology Dialysis Transplantation*.

[4] Fogo A. B. (2015). Causes and pathogenesis of focal segmental glomerulosclerosis. *Nature Reviews Nephrology*.

[5] Troost J. P., Waldo A., Carlozzi N. E. (2020). The longitudinal relationship between patient-reported outcomes and clinical characteristics among patients with focal segmental glomerulosclerosis in the nephrotic syndrome study network. *Clinical kidney journal.*.

[6] Rosenberg A. Z., Kopp J. B. (2017). Focal segmental glomerulosclerosis. *Clinical Journal of the American Society of Nephrology.*.

[7] Kawaguchi T., Imasawa T., Kadomura M. (2021). Focal segmental glomerulosclerosis histologic variants and renal outcomes based on nephrotic syndrome, immunosuppression, and proteinuria remission. *Nephrology Dialysis Transplantation*.

[8] Cheung A. K., Chang T. I., Cushman W. C. (2021). Executive summary of the KDIGO 2021 clinical practice guideline for the management of blood pressure in chronic kidney disease. *Kidney International.*.

[9] Beermann J., Piccoli M.-T., Viereck J., Thum T. (2016). Non-coding RNAs in development and disease: background, mechanisms, and therapeutic approaches. *Physiological Reviews*.

[10] Esteller M. (2011). Non-coding RNAs in human disease. *Nature reviews genetics.*.

[11] Denby L., Baker A. H. (2016). Targeting non-coding RNA for the therapy of renal disease. *Current opinion in pharmacology.*.

[12] Chen A., Liu Y., Lu Y., Lee K., He J. C. (2021). Disparate roles of retinoid acid signaling molecules in kidney disease. *American Journal of Physiology-Renal Physiology.*.

[13] Qi H., Fu J., Luan J. (2020). miR-150 inhibitor ameliorates adriamycin-induced focal segmental glomerulosclerosis. *Biochemical and biophysical research communications.*.

[14] Zhang C., Zhang W., Chen H.-M. (2015). Plasma microRNA-186 and proteinuria in focal segmental glomerulosclerosis. *American Journal of Kidney Diseases.*.

[15] Zhang C., Liang S., Cheng S. (2018). Urinary miR-196a predicts disease progression in patients with chronic kidney disease. *Journal of Translational Medicine*.

[16] Edgar R., Domrachev M., Lash A. E. (2002). Gene Expression Omnibus: NCBI gene expression and hybridization array data repository. *Nucleic acids research.*.

[17] Barrett T., Wilhite S. E., Ledoux P. (2012). NCBI GEO: archive for functional genomics data sets—update. *Nucleic Acids Research*.

[18] Consortium GO (2019). The gene ontology resource: 20 years and still GOing strong. *Nucleic Acids Research*.

[19] Kanehisa M., Furumichi M., Tanabe M., Sato Y., Morishima K. (2017). KEGG: new perspectives on genomes, pathways, diseases and drugs. *Nucleic acids research.*.

[20] Zhou Y., Zhou B., Pache L. (2019). Metascape provides a biologist-oriented resource for the analysis of systems-level datasets. *Nature Communications*.

[21] Szklarczyk D., Gable A. L., Lyon D. (2019). STRING v11: protein–protein association networks with increased coverage, supporting functional discovery in genome-wide experimental datasets. *Nucleic Acids Research*.

[22] Otasek D., Morris J. H., Bouças J., Pico A. R., Demchak B. (2019). Cytoscape automation: empowering workflow-based network analysis. *Genome biology.*.

[23] Chin C.-H., Chen S.-H., Wu H.-H., Ho C.-W., Ko M.-T., Lin C.-Y. (2014). cytoHubba: identifying hub objects and sub-networks from complex interactome. *BMC Systems Biology*.

[24] Bader G. D., Hogue C. W. (2003). An automated method for finding molecular complexes in large protein interaction networks. *BMC Bioinformatics*.

[25] Zhou G., Soufan O., Ewald J., Hancock R. E., Basu N., Xia J. (2019). NetworkAnalyst 3.0: a visual analytics platform for comprehensive gene expression profiling and meta-analysis. *Nucleic Acids Research*.

[26] Agarwal V., Bell G. W., Nam J.-W., Bartel D. P. (2015). Predicting effective microRNA target sites in mammalian mRNAs. *eLife*.

[27] Paraskevopoulou M. D., Georgakilas G., Kostoulas N. (2013). DIANA-microT web server v5. 0: service integration into miRNA functional analysis workflows. *Nucleic acids research.*.

[28] Chen Y., Wang X. (2020). miRDB: an online database for prediction of functional microRNA targets. *Nucleic acids research.*.

[29] Sticht C., De La Torre C., Parveen A., Gretz N. (2018). miRWalk: an online resource for prediction of microRNA binding sites. *PLoS One*.

[30] Vejnar C. E., Blum M., Zdobnov E. M. (2013). miRmap web: comprehensive microRNA target prediction online. *Nucleic acids research.*.

[31] Li J.-H., Liu S., Zhou H., Qu L.-H., Yang J.-H. (2014). starBase v2. 0: decoding miRNA-ceRNA, miRNA-ncRNA and protein–RNA interaction networks from large-scale CLIP-Seq data. *Nucleic acids research.*.

[32] Hommos M. S., De Vriese A. S., Alexander M. P. (2017). The incidence of primary vs secondary focal segmental glomerulosclerosis: a clinicopathologic study. *Mayo Clinic Proceedings*.

[33] Miao J., FPE V., Hogan M. C. (2021). Identification of genetic causes of focal segmental glomerulosclerosis increases with proper patient selection. *Mayo Clinic Proceeding*.

[34] Chen Y. M., Liapis H. (2015). Focal segmental glomerulosclerosis: molecular genetics and targeted therapies. *BMC Nephrology*.

[35] Meyrier A. (2011). Focal and segmental glomerulosclerosis: multiple pathways are involved. *Seminars in Nephrology*.

[36] Rota C., Morigi M., Cerullo D. (2018). Therapeutic potential of stromal cells of non-renal or renal origin in experimental chronic kidney disease. *Stem cell research & therapy.*.

[37] Raina R., Wang J., Sharma A., Chakraborty R. (2020). Extracorporeal therapies in the treatment of focal segmental glomerulosclerosis. *Blood Purification*.

[38] Wong A. K., Sealfon R. S. G., Theesfeld C. L., Troyanskaya O. G. (2021). Decoding disease: from genomes to networks to phenotypes. *Nature Reviews. Genetics*.

[39] De Vriese A. S., Sethi S., Nath K. A., Glassock R. J., Fervenza F. C. (2018). Differentiating primary, genetic, and secondary FSGS in adults: a clinicopathologic approach. *J Am Soc Nephrol.*.

[40] Yao T., Udwan K., John R. (2019). Integration of genetic testing and pathology for the diagnosis of adults with FSGS. *Clinical Journal of the American Society of Nephrology*.

[41] Menon R., Otto E. A., Hoover P. (2020). Single cell transcriptomics identifies focal segmental glomerulosclerosis remission endothelial biomarker. *Insight*.

[42] Luque Y., Lenoir O., Bonnin P. (2017). Endothelial Epas1 deficiency is sufficient to promote parietal epithelial cell activation and FSGS in experimental hypertension. *Journal of the American Society of Nephrology*.

[43] Bukosza E. N., Kornauth C., Hummel K., Schachner H., Gebeshuber C. A. (2020). ECM characterization reveals a massive activation of acute phase response during FSGS. *International Journal of Molecular Science*.

[44] Rhee H., Song S. H., Kwak I. S. (2012). An explorative analysis of secretory receptor for advanced glycation endproducts in primary focal segmental glomerulosclerosis. *Clinical and Experimental Nephrology*.

[45] Kim E. Y., Dryer S. E. (2021). RAGE and *α*V*β*3-integrin are essential for suPAR signaling in podocytes. *Biochimica et Biophysica Acta - Molecular Basis of Disease*.

[46] Suresh C. P., Saha A., Kaur M. (2016). Differentially expressed urinary biomarkers in children with idiopathic nephrotic syndrome. *Clinical and Experimental Nephrology*.

[47] Haddad G., Lorenzen J. M., Ma H. (2021). Altered glycosylation of IgG4 promotes lectin complement pathway activation in anti-PLA2R1-associated membranous nephropathy. *The Journal of Clinical Investigation*.

[48] Hamdan D., Robinson L. A. (2021). Role of the CX3CL1-CX3CR1 axis in renal disease. *American Journal of Physiology. Renal Physiology*.

[49] Panzer U., Steinmetz O. M., Stahl R. A., Wolf G. (2006). Kidney diseases and chemokines. *Current Drug Targets*.

[50] Furuichi K., Kaneko S., Wada T. (2009). Chemokine/chemokine receptor-mediated inflammation regulates pathologic changes from acute kidney injury to chronic kidney disease. *Clinical and Experimental Nephrology*.

[51] Bignon A., Gaudin F., Hémon P. (2014). CCR1 inhibition ameliorates the progression of lupus nephritis in NZB/W mice. *Journal of Immunology*.

[52] Vielhauer V., Berning E., Eis V. (2004). CCR1 blockade reduces interstitial inflammation and fibrosis in mice with glomerulosclerosis and nephrotic syndrome. *Kidney International*.

[53] Gao Z. G., Ding Y., Jacobson K. A. (2010). P2Y_13_ receptor is responsible for ADP-mediated degranulation in RBL-2H3 rat mast cells. *Pharmacological Research*.

[54] Esposito T., Rendina D., Aloia A. (2012). The melatonin receptor 1A (MTNR1A) gene is associated with recurrent and idiopathic calcium nephrolithiasis. *Nephrology, Dialysis, Transplantation*.

[55] Huang Y. S., Lu K. C., Chao T. K. (2018). Role of melatonin receptor 1A and pituitary homeobox-1 coexpression in protecting tubular epithelial cells in membranous nephropathy. *Journal of Pineal Research*.

[56] Huang Y., Lu K., He C., Chen A., Wu C. (2021). The MTNR1A mRNA is stabilized by the cytoplasmic hnRNPL in renal tubular cells. *Journal of Cellular Physiology*.

[57] Hishikawa A., Hayashi K., Itoh H. (2018). Transcription factors as therapeutic targets in chronic kidney disease. *Molecules*.

[58] Usui T., Morito N., Shawki H. H. (2020). Transcription factor MafB in podocytes protects against the development of focal segmental glomerulosclerosis. *Kidney International*.

[59] Ren J., Xu Y., Lu X. (2021). Twist1 in podocytes ameliorates podocyte injury and proteinuria by limiting CCL2-dependent macrophage infiltration. *Insight*.

[60] Endlich N., Kliewe F., Kindt F. (2018). The transcription factor Dach1 is essential for podocyte function. *Journal of Cellular and Molecular Medicine*.

[61] Zhou H., Cheruvanky A., Hu X. (2008). Urinary exosomal transcription factors, a new class of biomarkers for renal disease. *Kidney International*.

[62] Zhang H., Liang S., Du Y. (2018). Inducible ATF3-NFAT axis aggravates podocyte injury. *Journal of Molecular Medicine (Berlin, Germany)*.

[63] Nelson T., Velazquez H., Troiano N., Fretz J. A. (2019). Early B cell factor 1 (EBF1) regulates glomerular development by controlling mesangial maturation and consequently COX-2 expression. *J Am Soc Nephrol.*.

[64] Fretz J. A., Nelson T., Velazquez H., Xi Y., Moeckel G. W., Horowitz M. C. (2014). Early B-cell factor 1 is an essential transcription factor for postnatal glomerular maturation. *Kidney International*.

[65] Braun D. A., Sadowski C. E., Kohl S. (2016). Mutations in nuclear pore genes _NUP93_ , _NUP205_ and _XPO5_ cause steroid- resistant nephrotic syndrome. *Nature Genetics*.

[66] Tumelty K. E., Higginson-Scott N., Fan X. (2018). Identification of direct negative cross-talk between the SLIT2 and bone morphogenetic protein-Gremlin signaling pathways. *The Journal of Biological Chemistry*.

[67] Trionfini P., Benigni A. (2017). MicroRNAs as master regulators of glomerular function in health and disease. *J Am Soc Nephrol.*.

[68] Müller-Deile J., Dannenberg J., Schroder P. (2017). Podocytes regulate the glomerular basement membrane protein nephronectin by means of miR-378a-3p in glomerular diseases. *Kidney International*.

[69] Ramezani A., Devaney J. M., Cohen S. (2015). Circulating and urinary microRNA profile in focal segmental glomerulosclerosis: a pilot study. *European Journal of Clinical Investigation*.

[70] Gebeshuber C. A., Kornauth C., Dong L. (2013). Focal segmental glomerulosclerosis is induced by microRNA-193a and its downregulation of WT1. *Nature Medicine*.

[71] Tay Y., Rinn J., Pandolfi P. P. (2014). The multilayered complexity of ceRNA crosstalk and competition. *Nature*.

[72] Hu S., Han R., Shi J. (2018). The long noncoding RNA LOC105374325 causes podocyte injury in individuals with focal segmental glomerulosclerosis. *The Journal of Biological Chemistry*.

[73] Cui X., Fu J., Luan J. (2020). CircZNF609 is involved in the pathogenesis of focal segmental glomerulosclerosis by sponging miR-615-5p. *Biochemical and Biophysical Research Communications*.

[74] Grayson P. C., Eddy S., Taroni J. N. (2018). Metabolic pathways and immunometabolism in rare kidney diseases. *Annals of the Rheumatic Diseases*.

[75] Mitrofanova A., Molina J., Santos J. V. (2018). Hydroxypropyl-*β*-cyclodextrin protects from kidney disease in experimental Alport syndrome and focal segmental glomerulosclerosis. *Kidney International*.

